# High-Performance Computational Recognition of Communication Signals Based on Bispectral Quadratic Feature Model

This article has been retracted.

**DOI:** 10.1155/2022/2773492

**Published:** 2022-04-26

**Authors:** Yarong Chen, Rui Zhu, Jianxin Guo, Feng Wang

**Affiliations:** School of Information Engineering, Xijing University, Xi'an, Shaanxi 710123, China

## Abstract

In response to the problems in the signal identification of radiation sources during the communication process, the bispectral quadratic feature model is applied to the identification algorithm for communication signals. According to the signal eigenvalues obtained from the bispectrum of the diagonal slices in the radiation source signals, the eigenvalues of the bispectrum diagonal slices can be extended from the frequency domain to the complex plane through the chirp-z operation in this paper, and the relevant data are obtained based on the bispectrum quadratic feature model of the signals by using the separation rules corresponding to the extended Babbitt distance. The bispectral quadratic feature model method is used to establish a sparse observation model, and the communication signal processing problem can be transformed into an estimation problem of signal motion parameters through the construction of a parametric database. At the same time, the high-resolution distance of communication signals is tested, and the communication signals are estimated by using the variational inference method. Finally, practical cases are analyzed, and the results indicate that the algorithm proposed in this paper can be used to identify different types of communication signals in accordance with simulated and measured data in the processing of communication signals in various environments, which has the certain anti-interference capacity to noise, can improve the identification rate of communication signals, and has verified the effectiveness and practicality of the algorithm proposed in this paper.

## 1. Introduction

The identification of communication signals is one of the key means of the communication industry at present, and it has been widely used in all walks of life and in the military field. As carriers of information data transmission, signals contain the features of the radiation source, which can be used to achieve accurate identification and detailed analysis of the communication signal, obtain the communication radiation source bispectrum features, and provide a basis for the subsequent communication signal radiation source effective identification [1, 2]. At present, for the purpose of implementing accurate identification of communication radiation source signals, generally selected communication signal bispectral features should comply with the features of the time shift without changes, the size without changes, and the phase without changes. In the signal bispectrum analysis, based on compliance with the aforesaid conditions while also needing to maintain high noise immunity, it is widely applied in different industrial fields [3, 4]. As the bispectrum analysis process is relatively simple and the workload of operations is relatively small, it can maintain a high level of higher-order spectral analysis features. Hence, it is more extensively used in the field of communication signal processing to acquire the bispectral quadratic features of the signal complex diagonal tangent on the basis of in-depth rooted communication signal bispectral quadratic features. Due to the existence of different identification accuracy of different high-performance computing subpaths, the use of the bispectral quadratic feature model can be obtained in accordance with the feature vector of the communication signal in the results of high-performance computing. Finally, the results of the experiment indicate that the proposed method is practical for the secondary identification algorithm of the communication signal features using the baroclinic distance criterion [5, 6]. As the communication signal has the innate advantages of all-day real-time, long-range role, high resolution, and so on, it can be used on a large scale in many fields such as high-resolution processing, feature extraction, signal classification, and so on, and the use of transmitting bispectral quadratic feature model can increase the acquired high-distance resolution. At the same time, it can also shorten the features of the receiver transient bandwidth, complete hardware reduction, and according to the subpulse carrier, frequency sequence can effectively reduce the observation time while effectively improving the anti-interference performance of the communication signals. Communication signals mainly indicate the signals of different factors (noise, no role of the signal) fused together, and the transmission path is more complex [7–9]. Even if a higher function of the communication signal is used, the signal results that can be obtained are not ideal. Hence, it is not easy to obtain a physical feature of the initial signal. However, deconvolution is a method to obtain the original signal in accordance with the feedback from the fused signal. This method is extensively used in different fields such as communication, communication signals, speech, and medicine. One of the more technologically advanced methods at present is the variational difference recovery method proposed by Chan et al. This calculation uses a partial differential gradient projection method for the Lagrange multiplier term to minimize the difference [10–12]. Its advantages are fast convergence, stability, and so on, especially for signals with steep edges. With regard to the regular dynamic adaptive calculation method, the numerical value of the difference is compared accordingly.

The bispectral quadratic feature model algorithm is applied to the issue of high-performance computing identification and analysis of communication signals in this paper by converting the estimation of motion parameters of communication signal identification into the evaluation problem of identification and analysis of reconstruction. This method focuses on the effective synthesis of low signal-to-noise ratio HR-RP based on the parameters of the communication signal identification motion signal in the search interval. In this way, it can quickly implement the estimation of the motion parameter impact under the premise of solving the HRRP reconstruction error under a low signal-to-noise ratio to identify the local optimal value according to the population update speed and finally accomplish the accurate processing of the communication signal motion parameters.

## 2. Models and Algorithm

### 2.1. Bispectral Quadratic Feature Model

In accordance with the setting of the carrier frequency sequence of the communication signal, it is possible to obtain the results of the bispectral quadratic feature model in accordance with the complete step FM signal within [13, 14]. In this way, the whole stepper FM signal contains *N* pulses, while *M* pulses (*M* < *N*) are extracted according to the sequence.

As the signal carrier frequency sequence of the bispectral quadratic feature model is set to *f*_*sm*_=*f*_*c*_+*g*(*m*)Δ*f*, in which Δ*f* stands for the pulse bandwidth of the signal and *g* stands for a subset in the interval [0:*N* − 1], then the bandwidth of the bispectral quadratic feature model can be expressed as *B*=*N*Δ*f*. Through the detailed analysis, it can be known that the corresponding correlation accumulation time is no greater than the whole communication signal step FM signal. Then the carrier frequency sequence of the communication signal can be set in accordance with the environmental information so that it possesses the enhanced anti-interference capability of itself.

It is assumed that the communication signal transmits a total of *k*-th groups of sparse step frequency modulation (FM) signals, then the sparse step FM high-performance operation of the first group can be expressed as follows:

(1) $$\begin{array}{c} s_{1}\left(t\right)=\sum_{m=0}^{M-1}\text{rect}\left(\frac{t-mT_{R}-kMT_{R}}{T_{p}}\right)\cdot \exp\left(j\pi \gamma {\left(t-mT_{R}-kMT_{R}\right)}^{2}\right)\\ \cdot \exp\left(j2\pi f_{sm}\left(t-mT_{R}-kMT_{R}\right)\right), \end{array}$$

where $t=\hat{t}+mT_{R}+kMT_{R}\left(m=1,2,\ldots ,M\right)$ stands for the whole calculation time, $\hat{t}$ stands for the fast time, and tect(*u*) stands for the corresponding rectangular window. If the value of tect(*u*) is 1 when |*u*| ≤ 1/2, then the value of tect(*u*) will become 0, in which *γ* indicates the modulation frequency of the communication signal and *T*_*P*_ and *T*_*R*_ stand for the pulse width of the communication signal and the number of pulse repetition periods in turn, respectively.

If the communication signal contains multiple scattering points, then the coefficient of the backward scattering of the *p*(*p*=1,2,…, *P*) scattering point can be expressed as *σ*_*p*_, which constitutes the “Stop-Go” model. The corresponding time delay value *τ*_*p*_(*t*) of the scattering point *p* within the pulse of the communication signal can be left unchanged, and then there will be *τ*_*p*_(*t*) ≈ *τ*_*p*_(*t*_*m*,*k*_), *t*_*m*,*k*_=*mT*_*R*_+*kNT*_*R*_. At the same time, with regard to the scattering point of the communication signal, the *m*-th subpulse echo under the *k*-th group of sparse step FM high-performance operation can be expressed as follows:

(2) $$\begin{array}{c} s_{2}\left(\hat{t},m,k\right)=\sigma_{p}\text{rect}\left(\frac{\hat{t}-\tau_{p}\left(t_{m,k}\right)}{T_{P}}\right)\cdot \exp\left(j\pi \gamma {\left(\hat{t}-\tau_{p}\left(t_{m,k}\right)\right)}^{2}\right)\\ \cdot \exp\left(j2\pi f_{sm}\left(\hat{t}-\tau_{p}\left(t_{m,k}\right)\right)\right)+\varepsilon \left(\hat{t}\right), \end{array}$$

where *τ*_*p*_(*t*_*m*,*k*_)=2*R*_*P*_(*t*_*m*,*k*_)/*c*, *R*_*P*_(*t*_*m*,*k*_) stands for the instantaneous slope distance between the *p*-th scattering point and the communication signal emission signal, in which *c* is the speed of light and $\varepsilon \left(\hat{t}\right)$ indicates the additive noise. If the accumulation angle *θ*_*m*,*k*_ of the signal to be processed is reduced, *R*_*P*_(*t*_*m*,*k*_)=*R*(*t*_*m*,*k*_)+*x*_*p*_sin  *θ*_*m*,*k*_+*y*_*p*_, in which *R*(*t*_*m*,*k*_) stands for the instantaneous slope distance between the communication signal, (*x*_*p*_, *y*_*p*_) stands for the reference point by the instantaneous slope distance, and the scattering point *p* of the communication signal is denoted by the coordinate value in its plane. Thus, for a high-speed communication signal, the distance between the signal reference point and the communication signal at the time point *t*_*m*,*k*_ can be obtained as *R*(*t*_*m*,*k*_)=*τ*_*R*_+*v*_*R*_*t*_*m*,*k*_+1/2*a*_*R*_*t*_*m*,*k*_^2^, where *r*_*R*_ stands for the distance between the communication signal and the communication signal at the initial time, *v*_*R*_ stands for the radial velocity of the signal, and *a*_*R*_ stands for the radial acceleration of the communication signal. The time delay of the communication signal can be expressed as *τ*_*ref*_(*t*_*m*,*k*_)=2*R*_*ref*_(*t*_*m*,*k*_)/*c*, where $R_{ref}\left(t_{m,k}\right)=r_{R}+{\hat{v}}_{R}t_{m,k}+1/2{\hat{a}}_{R}t_{m,k}^{2}$. In general, the estimation of *v*_*R*_ and *a*_*R*_ can be obtained in the tracking phase of the communication signal. Then, for the echoes to be solved by line frequency modulation, it can be assumed that $\hat{f}=\gamma \left(\hat{t}-2R\left(t_{m,k}\right)/c\right)$; thus, the communication signalization is converted to the following equation:

(3) $$\begin{array}{c} s_{3}\left(\hat{f},m,k\right)=\sigma_{p}\text{rect}\left(\frac{\hat{f}}{\Delta f}\right)\exp\left(j\frac{4\pi }{c}\left(f_{sm}+\hat{f}\right)\Delta R\right)\exp\left(j\frac{4\pi }{c}\left(\Phi_{P}+\Phi_{B}\right)\right)+\varepsilon \left(\hat{f}\right), \end{array}$$

where Δ*R*=*x*_*p*_sin  *θ*_*m*,*k*_+*y*_*p*_ and Φ_*P*_ and Φ_*B*_ stand for the phase error due to interpulse translation of the communication signal and the phase error due to interpulse translation of the pulse string, respectively. Thus, Φ_*P*_ and Φ_*B*_ can be expressed as follows:

(4) $$\begin{array}{c} \left.\begin{array}{c} \Phi_{P}=\Phi_{1}+\Phi_{2},\Phi_{B}=\Phi_{3}+\Phi_{4}+\Phi_{5}\\ \Phi_{1}=m^{2}\left(\frac{1}{2}\Delta a_{R}f_{0}T_{R}^{2}+\Delta f\Delta v_{R}T_{R}+k\Delta f\Delta a_{R}MT_{R}^{2}+\frac{1}{2}\hat{f}\Delta a_{R}T_{R}^{2}\right),\Phi_{2}=m^{3}\left(\frac{1}{2}\Delta a_{R}\Delta fT_{R}^{2}\right)\\ \Phi_{3}=m\left(\begin{array}{c} f_{0}\Delta v_{R}T_{R}+k\Delta f\Delta v_{R}MT_{R}+k\Delta a_{R}f_{0}MT_{R}^{2}+\hat{f}\Delta v_{R}T_{R}+\\ \frac{1}{2}\Delta a_{R}\Delta f{\left(kMT_{R}\right)}^{2}+k\Delta a_{R}\hat{f}MT_{R}^{2} \end{array}\right)\\ \Phi_{4}=k\left(f_{0}\Delta v_{R}MT_{R}+\hat{f}\Delta v_{R}MT_{R}\right),\Phi_{5}=k^{2}\left(\frac{1}{2}\Delta a_{R}f_{0}{\left(MT_{R}\right)}^{2}+\frac{1}{2}\hat{f}\Delta a_{R}{\left(MT_{R}\right)}^{2}\right) \end{array}\right\}, \end{array}$$

where Δ*v*_*R*_ stands for the residual velocity; $\Delta v_{R}=v_{R}-{\hat{v}}_{R}$, in which Δ*a*_*R*_ stands for the residual acceleration; and $\Delta a_{R}=a_{R}-{\hat{a}}_{R}$. Φ_1_ stands for the *m* quadratic phase term, which will generate the primary flap spreading in the phase of distance synthesis of the communication signal. Φ_2_ stands for the tertiary phase term of *m*; the communication signal distance image is synthesized as an asymmetric paraflap; and then this term can usually be expressed in the order of 10^−4^. Hence, it can be neglected. Φ_3_ contains the coupling terms of both *m* and *k*, which will lead to a distance image shift and cause the bending of the envelope. Φ_4_ stands for the primary phase term of *k*, which causes an azimuthal shift in the image of the communication signal and can also be neglected. Φ_5_ stands for the quadratic phase term of *k*. The azimuthal pulse pressure will cause the main flap spreading of the communication signal. For the purpose of constructing the reconstruction algorithm with sparse HRRP efficiently, the echoes can be converted into discrete form. If the number of pulse sampling points of each communication signal is set to *N*_*r*_, which complies with $\bar{L}=M\cdot N_{r}$ at the same time, then the *k*-th group of echoes can be expressed as *s*_*k*_=[*s*_0,*k*_,…,*s*_*m*,*k*_,…,*s*_*M*−1,*k*_]_1×*L*_^*T*^, in which *s*_*m*,*k*_=[*s*_0,*m*,*k*_,…,*s*_*N*_*r*_−1,*m*,*k*_]_1×*N*_*r*__, *s*_*n*_*r*_,*m*,*k*_=exp(*j*4*π*/*c*(*f*_*sm*_+*n*_*r*_/*N*_*r*_Δ*f*)(Δ*R*+Δ*v*_*R*_*t*_*m*,*k*_+1/2Δ*a*_*R*_*t*_*m*,*k*_^2^))+*ε*(*n*_*r*_).

The remaining transmission process parameters of the communication signal are introduced into the database, and then the sparse observation model of the communication signal can be expressed as follows:

(5) $$\begin{array}{c} s_{k}=D_{k}\left(\Delta v_{R},\Delta a_{R}\right)\theta_{k}+n, \end{array}$$

where $D_{k}\left(\Delta v_{R},\Delta a_{R}\right)\in {\mathbb{C}}^{\bar{L}\times L}$ stands for the database matrix corresponding to the *n*-th echo, *L*=*N* · *N*_*r*_, *θ*_*k*_ ∈ *ℂ*^*L*×1^ stands for the HRRP corresponding to the *k*-th echo, and *n* stands for the noise vector. Thus, *d*_*l*_^*k*^ can be obtained as follows:

(6) $$\begin{array}{c} d_{l}^{k}\left(\Delta \hat{v},\Delta \hat{a}\right)=f_{l}⊙g_{k}⊙h_{k}, \end{array}$$

where ⊙ stands for the inner product, *f*_*l*_ stands for the *l*-th column of the database *F*, *F*=[*F*_0_,…,*F*_*M*−1_]_*L*×*L*_^*T*^, $g_{k}={\left[g_{0,k},\ldots ,g_{M-1,k}\right]}_{\bar{L}\times 1}^{T}$, and $h_{k}={\left[h_{0,k},\ldots ,h_{M-1,k}\right]}_{\bar{L}\mathrm{\times 1}}^{T}$.

In accordance with the *m*-th subpulse of the signal, it can be known that

(7) $$\begin{array}{c} F_{m}={\left[\begin{array}{ccc} W_{m}\left(0,1\right) & \cdots & W_{m}\left(0,L-1\right)\\ \vdots & \vdots & \vdots \\ W_{m}\left(N_{r}-1,0\right) & \cdots & W_{m}\left(N_{r}-1,L-1\right) \end{array}\right]}_{N_{r}\times L},\\ g_{m,k}={\left[g_{m,k}\left(0\right)\cdots g_{m,k}\left(N_{r}-1\right)\right]}^{T},g_{m,k}\left(n_{r}\right)=\exp\left(j\frac{4\pi }{c}\left(f_{sm}+\frac{n_{r}}{N_{r}}\Delta f\right)\Delta v_{R}t_{m,k}\right), \end{array}$$

(8) $$\begin{array}{c} h_{m,k}={\left[h_{m,k}\left(0\right)\cdots h_{m,k}\left(N_{r}-1\right)\right]}^{T},\\ h_{m,k}\left(n_{r}\right)=\exp\left(j\frac{\mathrm{2\pi}}{c}\left(f_{sm}+\frac{n_{r}}{N_{r}}\Delta f\right)\Delta a_{R}t_{m,k}^{2}\right). \end{array}$$

As the signal reconstruction method based on the bispectral quadratic feature model can operate on the real matrix, it can be expressed as follows according to equation (8):

(9) $$\begin{array}{c} y=\Phi \theta +\varepsilon . \end{array}$$

In accordance with expression (9), the probability map model is established by using the Gamma-Gaussian algorithm [15, 16]. If the acquired noise *ε* is Gaussian white noise with 0 mean, then the probability of the signal echo *y* thus obtained is also Gaussian distributed, and the probability of *ε* distributed with *y* can be obtained as follows:

(10) $$\begin{array}{c} p\left(\varepsilon \right)=N\left(\varepsilon |0,\alpha^{-1}I\right),\\ p\left(y|\theta ,\alpha \right)=N\left(y|\Phi \theta ,\alpha^{-1}I\right), \end{array}$$

where *α* stands for the noise accuracy. The Gamma-Gaussian prior is introduced to the sparse vector *θ*, and the following can be obtained:

(11) $$\begin{array}{c} p\left(\theta |\Lambda \right)=N\left(\theta |0,\Lambda^{-1}\right), \end{array}$$

where the accuracy matrix Λ=diag(*λ*_1_,…, *λ*_*d*_) stands for the dimensional diagonal array, in which *D* = 2*L*. The accuracy parameters *λ*_*d*_(*d*=1,…, *D*) and *α* comply with the Gamma distribution, and the following can be obtained:

(12) $$\begin{array}{c} p\left(\lambda_{d}\right)=\text{Gamma}\left(\lambda |v_{1},v_{2}\right),\\ p\left(\alpha \right)=\text{Gamma}\left(\alpha |v_{3},v_{4}\right). \end{array}$$

The product of the distributions according to the probability model can be obtained as follows:

(13) $$\begin{array}{c} p\left(y,\theta ,\Lambda ,\alpha \right)=p\left(y|\theta ,\alpha \right)p\left(\theta |\Lambda \right)p\left(\alpha \right)\prod_{d}p\left(\lambda_{d}\right). \end{array}$$

On the other hand, the posterior distribution of the random variables can be expressed as the joint distribution of the variables divided by the marginal distribution *p*(*y*), and thus, the following can be obtained:

(14) $$\begin{array}{c} p\left(\theta ,\Lambda ,\alpha |y\right)=p\frac{\left(y,\theta ,\Lambda ,\alpha \right)}{p\left(y\right)}. \end{array}$$

It is highly difficult to calculate the posterior distribution based on the model directly. Thus, high-performance computing is carried out to resolve the approximate posterior distribution so as to enable the HRRP synthesis under the low signal-to-noise ratio (SNR) conditions.

### 2.2. Identification of High-Performance Computing of Communication Signals

#### 2.2.1. Processing of Signals with Large Angle and Low Signal-to-Noise Ratio

In the research on the performance of communication signals, the parameters related to the communication signals are analyzed, with the main parameters as follows:

(1) Insertion loss (IL): The loss of signal power due to the addition of a device in a transmission line or fiber is denoted by decibels (dB). When the power transmitted to the load before insertion is P_in_ and at the same time the power received by the load after insertion is P_ℒ_, then the equation for insertion loss in dB can be obtained as follows:
  (15) $$\begin{array}{c} \text{IL}=10\;\log\frac{P_{\text{in}}}{P_{ℒ}}=-10\;\log\;\left(1-\left|\Gamma_{\text{in}}\right|\right), \end{array}$$
where |Γ_in_| stands for the reflection coefficient, which can be expressed as follows in accordance with the connection between IL and *𝒮*_21_:
  (16) $$\begin{array}{c} \text{IL}=10\;\log\frac{1}{{\left|S_{21}\right|}^{2}}=-10\;\log\;{\left|S_{21}\right|}^{2}. \end{array}$$
The relationship between P_ℒ_, P_in_, and *𝒮*_21_ in equation (16) is as follows:
  (17) $$\begin{array}{c} \frac{P_{\text{in}}}{P_{ℒ}}=\frac{1}{{\left|S_{21}\right|}^{2}}. \end{array}$$
(2) Bandwidth represents the selected range of the signal, that is, the width of the spectrum to be passed, the unit of the frequency range width, which is expressed in Hz, with the following equation:
  (18) $$\begin{array}{c} BW^{X\text{dB}}=f_{Η}^{XaB}-f_{L}^{X\text{dB}}. \end{array}$$
When the value of *X* is 3, 1, or 0.5, *f*_*H*_ and *f*_*L*_ stand for the frequencies on both sides of the passband when the reduction in the values of insertion loss on the left and right sides of the center frequency is *X* (dB).
(3) In-band fluctuation refers to the size of the fluctuation in the response amplitude of the passband, that is, the difference between the maximum and minimum values of the response amplitude. In the design process of communication signals, the smaller the in-band fluctuation, the better the performance of the communication signals.
(4) Return loss (RL) refers to the functional loss in the signal returned or reflected by the discontinuity in the transmission line. Discontinuity may not comply with the terminating load or the equipment inserted into the line, which is expressed in decibels (dB). The reflection system of the communication signal is also referred to as the reflection loss. The equation for return loss is as follows:
  (19) $$\begin{array}{c} \text{RL}=-10\;\log\;{\left[\frac{\text{VSWR}-1}{\text{VSWR}+1}\right]}^{2}. \end{array}$$
When VSWR represents the voltage standing wave ratio, the magnitude of the return loss is related to the standing wave ratio (VSWR) and the reflection coefficient (Γ). The increased return loss corresponds to a lower VSWR. Return loss is an index that measures how well the equipment matches the line. If the return loss is high, it means that the match is good. Generally, in the design of a communication signal, a high return loss and a low insertion loss mean that the performance of the communication signal is relatively good.
(5) VSWR refers to the value of the impedance matching between the load and the transmission line or waveguide. A larger value of the VSWR indicates a higher degree of matching. The VSWR stands for the ratio of the amplitude of the partial standing wave at the wave web (maximum value) to the amplitude of the node along the line (minimum value).
(6) The quality factor *Q* stands for the ability of the communication signal to allow separation of the neighboring frequencies in the signal, and its equation is as follows:
  (20) $$\begin{array}{c} Q=\frac{f_{o}}{\text{BW}}. \end{array}$$
When *f*_*o*_ represents the center frequency of the communication signal, BW stands for the 3 dB bandwidth. A larger value of *Q* indicates that the device has higher working stability, stronger frequency selectivity, lower loss, but narrower band; on the contrary, a smaller value of Q value indicates that the device's operating stability is lower, the frequency selectivity is weaker, the loss is relatively large, but the frequency band is wider. When the value of *Q* is increased in the design, the higher the Q value is, the stronger the performance of the device is.
(7) Resonant frequency: With regard to the communication signals, there are multiple ways to resolve the resonant frequency. Thus, there are also various factors affecting the resonant frequency. Common factors affecting the resonant frequency include the structure of the communication signals, the shape and the resonant mode, and so on. In practice, four methods are often used to resolve the resonant frequency: the electro-nano method, the total set parameter method, the field solution method, and the phase method.

The indicators mentioned above are used to measure the performance of a communication signal. In practice, it is not required to set the limit for all indicators, and some of the indicators can be optimized according to the actual demand.

#### 2.2.2. Processing Result of Measured Signals

The transfer function of a communication signal is a mathematical formula that expresses the frequency response features of the communication signal. With regard to the classical two-port communication signal, the transmission function equation is as follows:

(21) $$\begin{array}{c} |S_{21}{\left(jW\right)}^{2}|=\frac{1}{1+\varepsilon^{2}{ℱ}_{n}^{2}\left(\Omega \right)}, \end{array}$$

where *ε* stands for the ripple coefficient, ℱ_*n*_(Ω) stands for the functional characteristic of the low-pass prototype, and *Ω* stands for the frequency variable.

The features of communication signals are represented through the frequency response characteristics. With regard to the classification of communication signals as mentioned at the beginning of this paper, they can be divided into four types (i.e., low pass, high pass, band pass, and band resistance) according to the frequency response characteristics. The high pass, band pass, and band resistance can be obtained through the low-pass prototype of the frequency and components.

In the communication process, radiation source noise is mainly generated by the transmitter noise. In general, it refers to the amplitude of the communication signal, frequency, and pulse width and repetition frequency together causing abnormal changes, that is, the stability of the communication process signal resulting in radiation source noise. Signal instability can be roughly divided into two categories: regular instability and random instability. Regular instability is mainly due to inadequate power filtering, mechanical jitter, and so on; random instability is the noise generated by the transmitter tube and modulation pulse random jitter generated.

At present, the gradual improvement of communication signal protocol will help to improve the stability of transmitter. Thus, with the large-scale use of the main vibration amplification type of transmitter, the noise generated can mainly be divided into the following three aspects:

1. According to the amplitude frequency characteristics and phase frequency characteristics of the system, the cause of frequency-domain distortion can be analyzed.
2. The top of the modulated pulse generates vibration; the top begins to fall with the power supply fluctuations of the transmitter due to the signal corresponding to the parasitic phase or the amplitude caused by the time-domain distortion phenomenon.
3. The main control oscillator has insufficient frequency stability and phase stability. The different circuits or devices used for different communication transmitters result in different transmitter noises for various communications.

Hence, the uncoordinated modulation within the communication signal pulse is due to the transmitter noise. As the noise is generated due to various kinds of parasitic modulation. The communication signals present differences in signal features.

The noise output from the communication transmitter indicates more non-Gaussian and non-linear features, and in the bispectral analysis, the signal amplitude and phase information are maintained. At the same time, the effect of Gaussian non-color noise on non-Gaussian signals bispectrum is completely suppressed, which can be used for the extraction of unconscious modulation features. Thus, the following concept of bispectrum is obtained accordingly.

It is assumed that the high order cumulant *c*_*kx*_(*τ*_1_, *τ*_2_,…, *τ*_*k*−1_) is absolutely summable, that is, the following can be obtained:

(22) $$\begin{array}{c} \sum_{\tau_{1}=-\infty }^{\infty }\cdots \sum_{\tau_{k-1}=-\infty }^{\infty }\left|c_{kx}\left(\tau_{1},\ldots ,\tau_{k-1}\right)\right|<\infty . \end{array}$$

The *k*-th-order spectrum is defined as the (*k* − 1)-order discrete Fourier transform of the *k*-th-order cumulants, that is, the following can be obtained:

(23) $$\begin{array}{c} S_{kx}\left(\omega_{1},\omega_{2},\ldots ,\omega_{k-1}\right)=\sum_{\tau_{1}=-\infty }^{\infty }\cdots \sum_{\tau_{k-1}=-\infty }^{\infty }c_{kx}\left(\tau_{1},\ldots ,\tau_{k-1}\right)\times \;\exp\left[-j\left(\omega_{1}\tau_{1}+\cdots +\omega_{k-1}\tau_{k-1}\right)\right]. \end{array}$$

Thus, the bispectrum, that is, the third-order spectrum, can be defined as follows:

(24) $$\begin{array}{c} B_{x}\left(\omega_{1},\omega_{2}\right)=\sum_{\tau_{1}=-\infty }^{\infty }\sum_{\tau_{2}=-\infty }^{\infty }c_{3x}\left(\tau_{1},\tau_{2}\right)\exp\left[-j\left(\omega_{1}\tau_{1}+\omega_{2}\tau_{2}\right)\right]. \end{array}$$

The bispectrum of the signal including phase noise can be obtained from the bispectrum estimation. The discrete noise signal obtained by Scout is represented by *X*(*n*)=*s*(*n*)+*W*(*n*), where *w*(*n*) represents the Gaussian white noise signal, *s*(*n*) includes the signal of non-Gaussian noise output from the transmitter, and *w*(*n*) and *s* (*n*) are independent of each other. If the cumulative quantity is solved three times for *x*(*n*), the following can be obtained:

(25) $$\begin{array}{c} c_{3x}\left(\tau_{1},\tau_{2}\right)=E\left\{\left[s\left(n\right)+w\left(n\right)\right]\left[s\left(n+\tau_{1}\right)+w\left(n+\tau_{1}\right)\right]\left[s\left(n+\tau_{2}\right)+w\left(n+\tau_{2}\right)\right]\right\}. \end{array}$$

Equation (4) is expanded and combined to obtain the following:

(26) $$\begin{array}{c} c_{3x}\left(\tau_{1},\tau_{2}\right)=c_{3s}\left(\tau_{1},\tau_{2}\right)+c_{3w}\left(\tau_{1},\tau_{2}\right)+E\left[w\left(n\right)\right]\left[c_{2x}\left(\tau_{1}\right)+c_{2x}\left(\tau_{2}\right)+c_{2s}\left(\tau_{2}-\tau_{1}\right)\right]\\ +E\left[s\left(n\right)\right]\left[c_{2w}\left(\tau_{1}\right)+c_{2w}\left(\tau_{2}\right)+c_{2w}\left(\tau_{2}-\tau_{1}\right)\right]. \end{array}$$

As long as the mean value of the signal and noise is zero, the following can be obtained:

(27) $$\begin{array}{c} c_{3x}\left(\tau_{1},\tau_{2}\right)=c_{3s}\left(\tau_{1},\tau_{2}\right)+c_{3w}\left(\tau_{1},\tau_{2}\right). \end{array}$$

As *w*(*n*) is a Gaussian noise signal, *c*_3*w*_(*τ*_1_, *τ*_2_) can be excluded from the calculation. Thus, it can be known that the communication letter can be used to eliminate the white noise after the third-order accumulation, then the bispectrum can be determined by *c*_3*s*_(*τ*_1_, *τ*_2_), that is, the following can be obtained:

(28) $$\begin{array}{c} c_{3x}\left(\tau_{1},\tau_{2}\right)=c_{3s}\left(\tau_{1},\tau_{2}\right)=E\left\{s\left(n\right)s\left(n+\tau_{1}\right)s\left(n+\tau_{2}\right)\right\}. \end{array}$$

In accordance with the above analysis, it can be observed that the evaluated bispectral features are mainly composed of the features of the signal itself and non-Gaussian noise. Hence, the bispectrum in the communication signal is assessed mainly based on the features specific to the signal itself, and it is also possible to obtain the features specific to various communications.

However, if the two-dimensional function can adopt the full-duplex spectrum as the signal feature to produce a two-dimensional template for matching, the number of operations can be excessively high, which will not comply with the high standard requirements for signal radiation source identification. The key to solving this issue lies in the introduction of high-performance computing bispectrum; in equation (28), the two-dimensional bispectrum is converted into a one-dimensional function. However, the high-performance computing bispectrum has the following defects:

1. The implementation of high-performance computing bispectrum is often a high-performance computation along each path. However, the secondary features obtained by this mode of computation are not consistent for the results to be recognized, and some of the bispectral points have relatively less effect on the results of the recognized targets and are subordinate to the ordinary bispectrum.
2. If there is a cross-term in the initial observed signal, the high-order accumulation calculated by using the multi-correlation function will lead to the result that the cross-term becomes more complicated. As the cross-term is generated by a random distribution, it is impossible to eliminate the cross-term based on the determined calculation method.

For the purpose of extracting the secondary features of the bispectrum as the features of the bispectrum and eliminating or decreasing the defects that occur in the process of high-performance computation of the bispectrum, the characteristic parameters that are available for communication signals can be obtained with optimal separability in the secondary features of the bispectrum. As a result, it can effectively solve many problems such as cross-terms caused by ordinary bispectral points and high-performance computing.

In order to make the communication signal meet the actual performance characteristics, it is necessary to design an appropriate chamfer size in the design process. When the ring size becomes larger, the upper and lower passband edges move along the transmission zero point, and the attenuation pole becomes smaller. The intermediate frequency of the communication signal tends to be a higher frequency, which changes the frequency characteristics of the communication signal. With the shortening of the distance between patch resonances and the smaller the passband bandwidth, the attenuation point will first become smaller and then become larger. Therefore, HFSS software is used to optimize the structural parameters of the communication signal, and finally, the structural dimensions of the communication signal are obtained, as shown in Table 1.

By selecting a vector analysis instrument to test the communication signal, Figure 1 is the simulation test diagram corresponding to the communication signal. From Figure 1, it can be seen that the intermediate frequency of double passband communication signal is 3.8 GHz and 5.9 GHz, and the bandwidth corresponding to 3 dB is 13.5% and 6.2%, respectively. The minimum insertion loss in broadband is 0.7 dB and 1.3 dB in turn, and the return loss in the passband is not higher than 60 dB. In addition, there are zero points at the edges of the upper and lower passbands, which greatly improves the suppression characteristics of the stopband. The experimental data are in good agreement with the simulation data.

Since the conjugate prior is adopted in this paper for probabilistic modeling, the closed-form solution of the posterior distribution can be obtained directly by carrying out high-performance computing [17]. It is assumed that *X* stands for the observed data and *w* stands for the set of random variables; then the expression of the approximate posterior distribution can be obtained as follows:

(29) $$\begin{array}{c} \ln\;q\left(w_{j}\right)=E_{q_{i}\neq j}\left[\ln\;q\left(X,w\right)\right]+\text{const,} \end{array}$$

where const. stands for a constant that guarantees the normalization of the posterior distribution. In the subsequent section, in accordance with the equation (18) and the probability model established, the approximate posterior distributions of the variables *θ*, *α*, and Λ are solved for the sparse reconstruction by using the high-performance computing. In accordance with the mean field assumption, equation (14) is given in the form of the posterior multiplication of *θ*, *α*, and Λ.

(30) $$\begin{array}{c} p\left(\theta ,\Lambda ,\alpha |y\right)\approx q\left(\theta \right)q\left(\Lambda \right)q\left(\alpha \right)=q\left(\theta \right)\prod_{d}q\left(\lambda_{d}\right)q\left(\alpha \right). \end{array}$$

The steps for the *θ* solution are described as follows:

**Step 1 .**

Initialization. Given Φ, v1, v2, v3, v4, Λ, and *α* are initialized, the termination threshold is *η*_1_, and the number of terminations is G2.

**Step 2 .**

Update the variable *α*, and its approximate posterior distribution is the Gamma distribution according to equation (14), as shown in the following equation:

(31) $$\begin{array}{c} q\left(\alpha \right)=\text{Gamma}\left(\alpha |a^{\prime },b^{\prime }\right), \end{array}$$

where $a^{\prime }=v_{3}+\bar{L}/2$ and *b*′=*v*_4_+1/2*E*_*q*(*θ*)_ · [(*y* − Φ*θ*)^*T*^(*y* − Φ*θ*)], in which $\bar{L}$ stands for the length of *y*. At this point, the expectation of *α* can be obtained as follows:

(32) $$\begin{array}{c} E_{q\left(\alpha \right)}\left[\alpha \right]=\frac{a^{\prime }}{b^{\prime }}. \end{array}$$

**Step 3 .**

Update the variable Λ, and the approximate posterior distribution of the *d*-th element *λ*_*d*_ is the Gamma distribution, as shown in the following equation:

(33) $$\begin{array}{c} q\left(\lambda_{d}\right)=\text{Gamma}\left(\lambda_{d}|e_{d}^{\prime },f_{d}^{\prime }\right), \end{array}$$

where *e*_*d*_′=*v*_1_+1/2 and *f*_*d*_′=*v*_2_+1/2*E*_*q*(*θ*)_[*θ*_*d*_^2^]. Thus, the expectation of *λ*_*d*_ can be obtained as follows:

(34) $$\begin{array}{c} E_{q\left(\lambda_{d}\right)}\left[\lambda_{d}\right]=\frac{e_{d}^{\prime }}{f_{d}^{\prime }}. \end{array}$$

**Step 4 .**

Update the variable *θ*, and its approximate posterior distribution is the Gaussian distribution, as shown in the following equation:

(35) $$\begin{array}{c} q\left(\theta \right)=N\left(\theta |\mu {}^{\prime },\Sigma^{\prime }\right), \end{array}$$

where Σ′=(*E*_*q*(Λ)_[Λ]+*E*_*q*(*α*)_[*α*]Φ^*T*^Φ)^−1^ and *μ*′=*E*_*q*(*α*)_[*α*]Σ′Φ^*T*^*y*. At this time, the following can be obtained:

(36) $$\begin{array}{c} E_{q\left(\theta \right)}\left[{\left(y-\Phi \theta \right)}^{T}\left(y-\Phi \theta \right)\right]={\left(y-\Phi \mu {}^{\prime }\right)}^{T}\left(y-\Phi \mu {}^{\prime }\right)+\text{trace}\left(\Phi^{T}\Phi \Sigma^{\prime }\right). \end{array}$$

**Step 5 .**

Repeat Steps 2 to 4, and the iteration is suspended when the relative change of $\hat{\theta }$ from the previous estimate does not exceed the threshold value *η*_1_.

In the following section, the accuracy requirement for $\left(\Delta {\hat{v}}_{R},\Delta {\hat{a}}_{R}\right)$ is analyzed according to equation (4). With regard to the HRRP synthesis, the quadratic phase term Φ_1_ can lead to distance image spreading. Hence, it is required that the change in the coherent accumulation time Φ_1_ of the burst should be less than *π*/2. Thus, the following can be obtained:

(37) $$\begin{array}{c} \left|\Delta \hat{v}\right|\leq \frac{c}{8M^{2}\Delta fT_{R}},\\ \left|\Delta \hat{a}\right|\leq \frac{c}{4f_{0}M^{2}T_{R}^{2}}. \end{array}$$

In practice, equation (26) can usually be met. Hence, the effect of $\Delta \hat{a}$ on HRRP synthesis is neglected. For the purpose of eliminating the envelope bending caused by the first-order phase term field of Φ_3_, it is required that the envelope shift induced by the residual velocity and the residual acceleration during the processing observation time should not exceed the specified range. Thus, the following can be obtained:

(38) $$\begin{array}{c} \left|\Delta \hat{v}\right|\leq \frac{c}{4M\Delta f\left(KMT_{R}\right)},\\ \left|\Delta \hat{a}\right|\leq \frac{c}{2M\Delta f{\left(KMT_{R}\right)}^{2}}. \end{array}$$

It should be noted that the linear phase of $\Delta \hat{v}$ generated between the bursts leads to the shift and bending of the distance image and $\Delta \hat{a}$ results in the widening and scattering of the azimuthal main flap.

For the purpose of obtaining excellent azimuthal focus, it is required that the peak reduction of the azimuthal image caused by the residual acceleration during the processing observation time should be no more than 3 dB; then the following can be obtained:

(39) $$\begin{array}{c} \left|\Delta \hat{a}\right|\leq \frac{7c}{4f_{0}{\left(KMT_{R}\right)}^{2}}. \end{array}$$

Hence, azimuthal focusing requires higher accuracy of the acceleration estimation. Finally, for the purpose of obtaining a well-focused image, the signal residual velocity and the residual acceleration should comply with equations (36) and (37). The subsequent experiments indicate that the algorithm proposed in this paper can comply with the requirement for estimation accuracy.

## 3. Simulation Experiment and Analysis

In this paper, the effectiveness of the proposed parameter estimation algorithm in the transmission process and the high resolution processing algorithm is verified based on the simulation data. The echoes of the satellite scattering point model (as shown in Figure 2 below) are generated in accordance with the parameters set out in Tables 2 and 3. It is assumed that the residual velocity and residual acceleration of the signals are 9 m/s and 1 m/s^2^, respectively. The bispectral quadratic feature model contains a total of 128 bursts, and each burst contains 64 randomly selected pulses from 80 consecutive full-band pulses (waveform 1). Through the addition of the complex Gaussian white noise to the echo, the echo signal-to-noise ratio can be increased from 0 dB to 15 dB in 5 dB steps. For each signal-to-noise ratio, 25 independent trials with different noise states are carried out with the number of genetic algorithm populations set to 40 and the number of genetic terminations set to 20. The algorithm proposed in this paper is compared with the PSO algorithm based on the parametric database (algorithm 1). In the comparison, the distance image entropy is weighted with the average distance image entropy as a signal function in accordance with algorithm 1.

The variation of the signal residual velocity and the acceleration estimation errors with the change in the SNR are shown in Figure 3. It can be observed that the estimation error of algorithm 1 at a low SNR is relatively large and fails to comply with equations (26) and (27). This is caused by the relatively large reconstruction error based on the OMP algorithm at the low SNR conditions. With the increase in the signal-to-noise ratio, the estimation error of algorithm 1 is decreased. However, the estimation results still fail to comply with the accuracy requirements and can result in image scattering. Compared with algorithm 1, the algorithm proposed in this paper is robust at any signal-to-noise ratio conditions. In addition, the errors of the residual velocity and residual acceleration estimation are 1 × 10^−2^ m/s and 5 × 10^−3^ m/s^2^, respectively, which can meet the estimation accuracy requirements of equations (26) and (27). The superior performance of the proposed algorithm in the motion parameter estimation under the low signal-to-noise ratio conditions is attributed to the following aspect: (1) the Gamma-Gaussian prior-based reconstruction algorithm that can implement the reconstruction of HRRP with high accuracy and (2) the excellent global optimization capability of the genetic algorithm.

As the estimation error of algorithm 1 at the signal-to-noise ratio of 0 dB is excessively large that the focusing processing cannot be implemented, for the purpose of a fair comparison, the database is established here in accordance with the motion parameter estimates obtained based on the proposed algorithm; then the OMP, GD, and high-performance calculations are carried out to resolve equation (9); and the images thus obtained are shown in Figure 4. From Figure 4, it can be observed that the algorithm proposed in this paper corresponds to the processing results with clear contours, fewer false points, and a better focusing effect than the other methods. In particular, the proposed algorithm can be used to describe the details of the solar sail panel more properly. In addition, the image entropy corresponding to the three methods can be obtained as 0.3310, 0.2935, and 0.2915.

For the purpose of fully verifying the proposed algorithm put forward in this paper, the stability of the three algorithms is further compared. The signal identification effect in the presence of external interference is analyzed accordingly.  Figure 5 below shows the corresponding time-domain waveforms of the signals.

In the process of high-performance computing identification of communication signals, it is impossible to ensure that the reception length and quality of the target signals and the computing under a certain number of conditions can present the stability of features, which is taken as an essential evaluation criterion for the practicality of the algorithm. Excellent methods for feature value extraction should not be constrained by the number of training, and such methods should have good robust performance when they are applied. After taking this point into full consideration, the identification accuracy of the training samples by using the target experimental signals is studied accordingly. The number of signal samples in each segment contains 500 points. For each class, the number of signal test samples is set to 100, and the number of training samples is adjusted to 50, 100, 150, and 200, respectively. The experiment is carried out 30 times. The mean value and variance of the identification rates obtained based on the three methods are recorded in turn, which are shown in Table 4.

In the empirical testing, different modulation methods are used to increase the number of training samples as shown in Table 1, which has effectively improved the identification rate of the proposed algorithm. As a result, the identification performance starts to be stabilized. When the real number identification is compared by using the three methods, the method proposed in this paper has the highest identification rate for the real signals measured, followed by the ISIB method, and the BSB method is the least effective. When *N*_*r*_ is increased from 50 to 200, the identification rate of the distance selected bispectrum of the BAS is improved by about 4%, while the ISIB and the method proposed in this paper show the improvement of about 3% and 2%, respectively. The results of the experiment indicate that the algorithm put forward in this paper has excellent stability, the identification results are less affected by the number of training samples, and the model thus established has good robustness, which suggests that the proposed algorithm has relatively strong practicality.

## 4. Conclusion

On the basis of the research on the fine features in the bispectral analysis of individual identification of radiation sources, the bispectral secondary features extracted are optimized by using the extended Babbitt distance criterion in accordance with the in-depth analysis of the bispectral features of communication signals diagonally sliced. This method can be used to implement the bounded deviation and identify the observation error values quickly and perform the complexity calculation of variational parameters effectively. The experiments indicate that the method is effective. The information on the original signals can also be recovered in a low signal noise background. The statistical features of communication scattering points and noise are used. Through practical analysis, the experimental results indicate that the method proposed in this paper has reduced the usage time. In addition, it can be applied to multiple types of communication signals. The bispectral features thus obtained always have excellent robustness at a low signal-to-noise ratio (SNR). When the signal-to-noise ratio is 0, the identification rate of high-performance computing of communication signals can achieve more than 90%. However, in general, a series of individual identification methods based on bispectral analysis have the common issue of a relatively low identification rate. Taking into account the subtle features in the other aspects of the signals, a feature vector is formed, which can further improve the practical effectiveness of the algorithm proposed in this paper.

## Figures and Tables

**Figure 1:** Simulation change diagram of communication signal.

**Figure 2:** Distribution of the signal scattering points.

**Figure 3:** Variation curve of the velocity acceleration estimation error with the change of SNR: (a) velocity estimation error and (b) acceleration estimation error.

**Figure 4:** Processing results of the simulation data waveform 1: (a) OMP, (b) GD, and (c) VBI.

**Figure 5:** Time-domain waveform of the actual measured signal.

**Table 1:** Structural parameters of level 1 UNICOM signal.

Structural parameters	Size (mm)
*a*	24
*b*	3
*c*	9
*d*	5
*e*	3
*f*	1.77
*g*	1.5
*L*	2

**Table 2:** Comparison of the operation complexity.

Reconstruction algorithm	OMP	GD	BQCM
Operational complexity	*𝒪*(*k*_0_*L*^2^)	*𝒪*(*L*^3^)	*𝒪*(*L*^3^)

**Table 3:** Parameters of the communication signal system.

(GHz) *f*_*c*_	PRF (KHz)	*T*_*R*_	B (MHz)	Δ*f*
10	6.4	20 ms	800	10 MHz

**Table 4:** Effect of different sample sizes on the identification results based on the three methods.

Experimental signal	*N*_*r*_ number	BSB		ISIB		Method put forward in this paper	
		Mean value (%)	Variance (10^−4^)	Mean value (%)	Variance (10^−4^)	Mean value (%)	Variance (10^−4^)
1, 2, 3, 4, 5	50	73.05	14.41	81.04	4.48	85.02	3.62
	100	74.65	8.36	81.21	3.98	86.06	2.38
	150	76.68	4.21	83.75	2.62	86.75	1.32
	200	77.15	6.53	84.27	3.14	87.21	1.54

## Data Availability

The data used to support the findings of this study are available from the corresponding author upon request.
